The article "Myogenic differentiation of VCP disease-induced pluripotent stem cells: A novel platform for drug discovery" was retracted in 2026. Reasons: errors in the images; duplicated images; overlap with earlier publications; original data or images not available.

# Myogenic differentiation of VCP disease-induced pluripotent stem cells: A novel platform for drug discovery

**DOI:** 10.1371/journal.pone.0176919

**Published:** 2017-06-02

**Authors:** Katrina J. Llewellyn, Angèle Nalbandian, Lan N. Weiss, Isabela Chang, Howard Yu, Bibo Khatib, Baichang Tan, Vanessa Scarfone, Virginia E. Kimonis

**Affiliations:** 1 Division of Genetics and Genomic Medicine, Department of Pediatrics, University of California-Irvine School of Medicine, Irvine, California, United States of America; 2 Sue and Bill Gross Stem Cell Research Center, University of California-Irvine School of Medicine, Irvine, California, United States of America; Indian Institute of Science Education and Research, INDIA

## Abstract

Valosin Containing Protein (VCP) disease is an autosomal dominant multisystem proteinopathy caused by mutations in the *VCP* gene, and is primarily associated with progressive muscle weakness, including atrophy of the pelvic and shoulder girdle muscles. Currently, no treatments are available and cardiac and respiratory failures can lead to mortality at an early age. VCP is an AAA ATPase multifunction complex protein and mutations in the *VCP* gene resulting in disrupted autophagic clearance. Due to the rarity of the disease, the myopathic nature of the disorder, ethical and practical considerations, VCP disease muscle biopsies are difficult to obtain. Thus, disease-specific human induced pluripotent stem cells (hiPSCs) now provide a valuable resource for the research owing to their renewable and pluripotent nature. In the present study, we report the differentiation and characterization of a VCP disease-specific hiPSCs into precursors expressing myogenic markers including desmin, myogenic factor 5 (MYF5), myosin and heavy chain 2 (MYH2). VCP disease phenotype is characterized by high expression of TAR DNA Binding Protein-43 (TDP-43), ubiquitin (Ub), Light Chain 3-I/II protein (LC3-I/II), and p62/*SQSTM1* (p62) protein indicating disruption of the autophagy cascade. Treatment of hiPSC precursors with autophagy stimulators Rapamycin, Perifosine, or AT101 showed reduction in VCP pathology markers TDP-43, LC3-I/II and p62/*SQSTM1*. Conversely, autophagy inhibitors chloroquine had no beneficial effect, and Spautin-1 or MHY1485 had modest effects. Our results illustrate that hiPSC technology provide a useful platform for a rapid drug discovery and hence constitutes a bridge between clinical and bench research in VCP and related diseases.

## Introduction

Hereditary Inclusion Body Myopathy, Paget Disease of Bone, Frontotemporal Dementia (IBMPFD) and Amyotrophic Lateral Sclerosis (ALS), recently termed VCP-associated disease (VCP disease) is a multisystem disorder with a diverse collection of manifestations caused by mutations in the *valosin containing protein (VCP)* gene [1–4]. Inclusion body myopathy (IBM) is the most common feature present in up to 90% of affected individuals with an age of onset typically in their 30s. Patients typically demonstrate progressive weakness and atrophy of the skeletal muscles, generally starting with the pelvic and shoulder girdle muscles. Progressive muscle weakness typically advances to involve other limbs and respiratory muscles, resulting in patient mortality from cardiomyopathy or respiratory failure between approximately 40–60 years of age. Hallmarks of the muscle pathology include rimmed vacuoles, ubiquitin- and TDP-43-positive inclusions and increased autophagy markers such as Light Chain 3-I/II (LC3-I/II) and p62/*SQSTM1*. The second most common pathology is Paget’s disease of the bone (PDB) which is observed in 49% of patients [3, 5, 6], typically with onset in their 30s to 40s. PDB is caused by excessive osteoclastic activity and increased bone turnover and susceptibility to deformities like bowing and fractures [7–9]. The third most common component of VCP disease is frontotemporal dementia (FTD), with an average age of onset of 54 years with an overall frequency of 33% [1, 5, 10]. Hallmarks of the muscle and brain pathology include inclusions of ubiquitin and TDP-43 also seen in other proteinopathies associated with FTD [11–13]. Additional pathology manifestations of VCP mutations include ALS in up to 15% of VCP disease patients, with Parkinson’s disease (PD) [14] Alzheimer’s disease (AD) [15, 16], and cardiomyopathy among other associated manifestations [5]. Interestingly VCP mutations also account for 3% of isolated familial ALS (fALS) [17, 18]. Over 40 VCP mutations have been identified worldwide in families from several parts of the world including Germany [19, 20], France [21], Austria [22], Italy [23], the United Kingdom [24], Australia [25], Korea [26], and the United States [1, 2, 5, 6, 27–31], with the R155H mutation present in more than 50% of affected individuals.

On a molecular level, VCP, a member of the type II AAA+ ATPase family, plays an important role in a plethora of cellular activities and recent studies have implicated the ubiquitin proteasome protein degradation pathway [32, 33], the autophagy cascade [5, 30, 33, 34], mitochondrial quality control [32, 35–37] and potentially other signaling pathways in the pathogenesis of VCP disease. *Sequestosome 1* (p62/*SQSTM1*) interacts with Light Chain 3 (LC3-I/II), which is an autophagic effector protein, to facilitate the process of autophagic uptake of aggregated proteins [5]. VCP is necessary to initiate the retro-translocation process for misfolded endoplasmic reticulum (ER) proteins; thus, mutations in the VCP gene result in defective ER associated protein degradation (ERAD) and ER stress responses [28]. Although VCP disease is a relatively rare disorder, exploration of its cellular and molecular mechanisms holds promise for explaining shared pathologies of more common proteinopathies, such as ALS, PD, and FTD.

Stem cells have revolutionized the field of human cell culture because they provide an immortal population of pluripotent cells, which can theoretically differentiate into any cell type [38–40]. Due to their renewable and pluripotent nature, stem cells also allow for the development of therapies for rare muscle conditions such as VCP disease, where tissue is sparse or difficult to access. In particular, patient-specific induced pluripotent stem cells (iPSCs) represent an excellent tool for modeling disease since they can be generated from adult somatic cells, thus, avoiding the ethical considerations involved with using embryonic stem cells. iPSCs will continue to be a sustainable method to model disease for gene therapies, drug therapies, and for transplantable stem cells for neuromuscular and related diseases [38, 41–45]. iPSC technology is already being utilized in other neurodegenerative diseases, including ALS [46], Duchenne muscular dystrophy (DMD) [47], PD [48], AD [49, 50], macular degeneration [51, 52], and type I diabetes mellitus [53, 54]. Therefore, creation and characterization of human derived VCP disease iPSCs has offered a novel therapeutic platform to investigate mechanisms of VCP disease and further the development of effective treatment [55]. Differentiating these patient-derived iPSCs into a myogenic lineage has the promise to make significant contributions to our understanding of VCP disease [46, 47, 56–58]. The use of adult myogenic stem cells as a cell therapy for skeletal muscle regeneration has been attempted for decades, with only moderate success [40, 59–63]. However, several studies have recently reported development of more effective differentiation protocols with the use of skeletal muscle specific media and the induction of PAX3/7 with a retrovirus [47, 56, 64–69].

In this report, we differentiated patient-derived human induced pluripotent stem cells (hiPSC) into myogenic lineages to provide a useable resource to study the underlying pathological mechanisms of VCP disease and as a novel platform for a rapid drug screening. We showed a significant success rate of patient-derived and control iPSC differentiation into the myogenic lineages. Characterization of the VCP disease phenotype in our myogenic lineages revealed higher protein expression levels of classic VCP pathology including autophagy markers LC3-I/II, p62/*SQSTM1*, ubiquitin and upregulation and translocation of TDP-43 to the cytoplasm. We next screened the effects of various autophagy-modifying compounds to understand the molecular dysfunction in VCP pathology and as a therapeutic strategy for VCP-associated diseases. We observed significant improvement in pathology with autophagy inducers Rapamycin, Perifosine and AT101. Conversely chloroquine an autophagy inhibitor showed no benefit. Interestingly, Spautin-1 and MHY1485 showed a modest beneficial effect in preventing TDP-43 translocation from the nucleus to the cytoplasm. In summary, our study provides a unique and novel platform for investigating the underlying pathophysiology mechanisms of VCP disease and for rapid screening of new drugs that ameliorate autophagy dysfunction thus improving muscle integrity and/or slowing down the progression of muscle wasting in patients with VCP and related neurodegenerative diseases.

## Materials and methods

### Ethics statement

The University of California Irvine (Irvine, California) Institutional Review Board (IRB) (#2009–1005) approved this study including the consenting procedure. We explained the research to the participant, reviewed the consent form and provided an opportunity to ask questions in order to ensure that the subject understood the research. The subjects signed the approved consent form. Skin biopsy samples were submitted to Coriell repository and were used for the iPSCs generation. The control iPSCs were obtained from the University of Connecticut repository.

### Differentiation of iPSC into skeletal muscle lineage

VCP disease and control iPSCs were differentiated into skeletal muscle lineages using a modified protocol adapted from *Awaya et al*. (2012) [57]. Briefly, iPSCs were grown in mouse embryonic fibroblast (MEF) conditioned media (CM) supplemented with basic fibroblast growth factor (bFGF) (CM-bFGF) [70]. Once confluent, iPSCs were treated with 1 mg/mL collagenase in DMEM/F12 at 37°C for 5 min and removed from the plate by mechanical scraping. The cell clusters were then left floating in CM-bFGF for 7 days in a non-adhesive flask to form embryoid bodies (EBs). Next, the EBs were transferred to 0.2% gelatin-coated tissue culture plates in ITS medium (DMEM, 1X ITS-X (ThermoFisher Scientific, Carlsbad, CA), non-essential amino acids (ThermoFisher Scientific GlutamaxH supplement (ThermoFisher Scientific), and 100 mM 2-mercaptoethanol for 14 days to promote a mesenchymal lineage [57]. To encourage skeletal muscle differentiation, the medium was changed to skeletal muscle induction medium skIM (SkIM: high-glucose DMEM supplemented with 10% fetal calf serum (FCS; ThermoFisher Scientific), 5% horse serum (HS; Sigma, St. Louis, MO), non-essential amino acids (Invitrogen), and 100 mM 2-mercaptoethanol for 7 days [57]. The differentiated cells were analyzed on days 7, 21, 49, 56, 63, and 70. Images of differentiation by differential interference contrast (DIC) microscopy were taken on days 0, 21, 50, 69. Primary myoblasts from the same patient or control subjects were used in this investigation for comparison of morphology.

### Flow cytometry

Differentiated myoblasts were phenotyped and sorted by flow cytometry (Sue and Bill Gross Stem Cell Institute, University of California-Irvine, Irvine, CA). Briefly, myogenic precursors at days 35 and 49 were dissociated with dissociation buffer (ThermoFisher Scientific) and stained with cell surface pluripotency marker, anti-CD34, and mesenchymal stem cell (MSC) markers anti-CD73, anti-CD105 and anti-CD29 (Life Technologies) and skeletal muscle marker, anti-CD56 (ThermoFisher Scientific) as well as isotype controls (BD Pharmingen). Dead cells were excluded by propidium iodide (Sigma-Aldrich) and samples were analyzed using FACSAria II and FACS Diva software (BD Biosciences, Franklin Lakes, NJ).

### Treatments with autophagy-modifying agents

Day 50 myogenic progenitor patient and control cells were seeded onto gelatin-coated 4-well chamber slides or 6-well plates and cultured in sKiM media. Patient and control cells were either treated with autophagy inducers, Rapamycin (10 μM) [71, 72], Perifosine (also known as KRX-0401) (80 μM) [73] or AT101 (10μM) [74, 75] or autophagy inhibitors chloroquine (10 μM) [76, 77], Spautin-1 (10 μM) [78] or MHY1485 (2 μM) [79] for 24 hours. Following treatment, immunocytochemical and Western blot analysis were performed and analyzed.

### Immunocytochemical analysis

Myogenic progenitor cells were seeded, at days 21 and 50 onto gelatin-coated 4-well chamber slides and cultured in sKiM media. Cells were washed with PBS then fixed in 4% paraformaldehyde (PFA) for 15 minutes, and permeabilized with Triton X-100 for ICC staining. To check for pluripotent markers, cells were stained with anti-Oct-3/4 and Nanog (Sigma-Aldrich, St. Louis, MO). To check for myogenic differentiation, both early (anti-MYF-5, desmin and anti-PAX-7) and late stage markers (anti-MyoD and anti-MYH2) were used. For VCP disease pathology analysis, cells were taken at day 50 and seeded as aforementioned. Both treated and untreated cells were then stained for ‘classic’ VCP pathology markers, anti-TDP-43, p62*/SQSTM1* and LC3 (Abcam, Cambridge, MA).

### Western blot analysis

Protein samples from patient and control myogenic progenitors were extracted using RIPA buffer according to manufacturer’s instructions (Thermo Scientific, Rockford, IL). Protein concentrations were identified using the Nanodrop technique according to the manufacturer’s protocols. Equal amount of proteins from samples were run on Bis-Tris 4–12% NuPAGE gels using the Novex Mini Cell (Invitrogen Life Technologies, Carlsbad, CA). To confirm differentiation, both pluripotent markers (rabbit monoclonal anti-NANOG and rabbit monoclonal anti-Oct3/4) and myogenic markers (rabbit monoclonal anti-MYF-5, rabbit polyclonal anti-desmin, rabbit monoclonal anti-MyoG, rabbit polyclonal anti-MyoD and rabbit monoclonal anti-MYH2) were analyzed. To analyze expression levels of ‘classic’ VCP pathology, rabbit monoclonal anti-TDP-43, rabbit monoclonal anti-mTOR, rabbit monoclonal anti-LC3-I/II, rabbit monoclonal anti-p62/SQSTM1, and rabbit monoclonal anti-ubiquitin-specific antibodies were used. Equal protein loading was confirmed by rabbit monoclonal anti-GAPDH antibody staining. All antibodies were purchased from Abcam. Cytoplasmic and nuclear protein factions were extracted using NE-PER kit (Thermo Scientific). Densitometry was performed to quantitate the Western blot bands using Image J Program (National Institutes of Health, Bethesda, MD).

### Statistical analysis

Statistical analysis of densitometry data of three Western blot trials was performed using SPSS standard software (Version 13.0. Chicago, SPSS Inc.). Two-tailed student’s *t* test was used to calculate *p* values.

## Results

### Differentiation and validation of control and patient iPSC-derived myogenic lineage

Our goal in this study was to establish efficient differentiation of human iPSCs into a myogenic lineage to model VCP disease and related neuromuscular diseases. Additionally, we aimed to utilize these cells in subsequent drug screening studies. A schematic of human iPSC differentiation and maturation into myotubes is depicted in Fig 1A. We first cultured and imaged differentiation of iPSCs (Day 0–69) into a myogenic lineage in patient (Fig 1B) and control iPSC (Fig 1D) lines shown by differential interference contrast (DIC) microscopy. By day 69, these cells closely resembled primary myoblasts taken from the same patient (Fig 1C) or control myoblasts (Fig 1E).

**Fig 1:** Differentiation of patient and control VCP iPSC into myogenic lineages. (A) Schematic of early hiPSCs and embryoid bodies commitment (Days 0–50) into early mesenchymal stem/stromal cells (MSC) and differentiation into myoblasts (Day 64). (B) Myogenic differentiation of human iPSC at Days 0, 21, 50, and 69 with (C) primary myoblast cells from a 57-year old patient diagnosed with IBMPFD. (D) Control derived myogenic precursors at Days 0, 21, 50, and 69 with (E) primary myoblast cells from age matched healthy control. Differential interference contrast (DIC) microscopy images of differentiated primary mature myoblasts from iPSCs. Scale: Bar = 1000 μm.

Subsequently, myoblast lineages differentiated from patient-derived inducible pluripotent stem cells (iPSCs) were validated using both immunohistochemical (IHC) and Western blot methods. Staining with early myogenic precursor markers such as MYF-5, desmin, and Pax7 illustrated increased expression from day 21, and they are still expressed at day 50 (Fig 2A). Interestingly, late myogenic skeletal markers, such as MyoD and MYH2 were expressed by day 50, however, not detected at earlier time points (Fig 2B). Western blot analysis revealed the cells had lost expression of their pluripotent marker (Oct3/4 and Nanog) after day 21. Myogenic precursor markers (desmin, MYF5 and MyoD) begin to be expressed starting on day 21 and continue through day 50. Late myogenic markers (MyoG and MYH2) begin to be expressed last at day 50 (Fig 2E). Myogenic differentiation was then validated by FACS analysis using the pluripotent marker (CD34: 96.6% negative) and myoblast marker (CD56: 92.3% positive). Similarly, these cells were also positive for MSC markers (CD73, CD29 and CD105) (Fig 2F).

**Fig 2:** Validation of myogenic differentiation in patient and control-derived iPSCs. Human iPSC from a 57-year old patient diagnosed with VCP disease-derived myogenic precursors were stained at Day 21 and Day 50 with (A-B) MYF-5, desmin, and Pax7; (C-D) MyoD and MYH2. Representative merged overlay images of stained iPSC with DAPI. Scale: Bar = 50 μM. (E) Western blot analysis of myoblast differentiation markers at Day 0, 7, 21, 35, and 50 with anti-Oct3/4, Nanog, desmin, MYF5, MyoD, MyoG and MYH2. GAPDH was used as a positive loading control. (F) FACS analysis of iPSC-derived MSCs with pluripotent marker (CD34) and myoblast marker (CD56). (G) CD34 isotype control. (H) CD65 isotype control.

### Accumulation of autophagy markers in differentiated hiPSC myogenic lineage

The autophagy cascade whereby long-lived proteins are degraded is of critical importance in understanding the possible underlying mechanisms in VCP disease. We and others have previously shown that the autophagic pathway is disrupted in patients’ myoblasts and in VCP^R155H/+^ mouse models [30, 80, 81]. To determine the pathophysiological effects of *VCP* mutations on our differentiated disease myogenic lineages, we stained with mAbs specific to TDP-43, a hallmark of VCP pathology, mTOR, and autophagy markers LC3-I/II and p62/*SQSTM1*. Compared to the control myoblasts, VCP myoblasts showed increased cytoplasmic staining of TDP-43, (Fig 3A and 3B) and increased protein expression levels of the autophagic markers, LC3-I/II and p62/*SQSTM1*, thereby suggesting impaired degradation of the proteins involved in the autophagosome-lysosomal cascade (Fig 3A and 3B). Western blot analysis and densitometry analysis of Western blot data relative to GAPDH, confirmed these results with significant increased TDP-43 (p<0.001, both day 21 and 50), LC3I/II (p<0.005 on day 21, p<0.001 on day 50), p62/*SQSTM1* (p<0.001, both day 21 and 50) and ubiquitin (p<0.001, both day 21 and 50) (Fig 3C and 3D) as well as the cytoplasmic mislocalization of TDP-43 in VCP myoblasts (Fig 3E).

**Fig 3:** Characterization of autophagy signaling cascade in control and patient VCP iPSC-derived myoblast lineages. Differentiated (A) control and (B) iPSC-derived myoblast lineages were immunostained with TDP-43, LC3, and p62/*SQSTM1*. Representative merged overlay images of stained iPSC with DAPI. Scale: Bar = 50 μM. (C) Western blot analysis of iPSC-derived control and patient myoblasts with anti-TDP-43, LC3I/II, p62/*SQSTM1*, and ubiquitin. GAPDH was used as a positive loading control. (D) Densitometry analyses confirmed these Western blot results. Statistical significance is denoted by *p<0.05, **p<0.005 and ***p<0.001. (E) Western blot analysis of cytoplasmic (Cy) and nuclear (Nu) factions of iPSC-derived control and patient myoblasts with anti-TDP-43.

### Autophagy modifiers and VCP's interplay in the autophagy cascade

Several studies showed that the autophagy cascade is highly dysregulated in VCP disease [30, 82–84]. However, the underlying mechanisms of such dysregulation remain to be fully elucidated. We, therefore, decided to utilize our differentiated patient-derived hiPSCs together with several autophagy inhibitors and activators that interact as various different points in the autophagy cascade (Fig 4A) to gain insight in the pathogenesis and explore if autophagy modulation could ameliorate VCP disease pathology. These modifiers and the location of their impact within the autophagy cascade are illustrated in Fig 4A.

**Fig 4:** Drug screening with autophagy inducers Rapamycin, Perifosine and AT101 in patient VCP iPSC-derived myogenic lineages. (A) Schematic of intervention with autophagy modifying agents. Green arrows show the active location of autophagy activators Rapamycin, Perifosine and AT101. Red arrows show the active location of autophagy inhibitors chloroquine, Spautin-1 and MHY1485. VCP is indicated to have an interactive role with Akt and as a chaperone protein with ubiquitin. (B) Untreated differentiated control and (C) untreated patient derived myogenic lineages. Patient derived myogenic lineage were treated with either (D) Rapamycin (10 μM), (E) Perifosine (80 μM) or (F) AT101 (10 μM) for 24 hours. Subsequently, cells were stained with TDP-43, LC3 or p62/*SQSTM1* antibodies. Representative merged overlay images of stained iPSC with DAPI. Scale: Bar = 25 μm. White dotted lines represent areas of increased or decreased expressions. (G) Western blot analysis of iPSC-derived control (C) and patient (P) myoblasts with mTOR, TDP-43, LC3I/II and p62/*SQSTM1*. GAPDH was used as a positive loading control. (H) Densitometry analyses of the Western blot. Black dotted line indicates expression over baseline control sample. Statistical significance is denoted by *p<0.05, **p<0.005 and ***p<0.001.

### Drug screenings with autophagy-modifiers

To explore the effects of autophagy-modifying drugs on the iPSC-derived patient VCP myoblasts, we treated them with autophagy stimulators Rapamycin, Perifosine, and AT101 (Fig 4) and autophagy inhibitors chloroquine, Spautin-1, and MHY1485 (Fig 5). These autophagy modifiers were selected to help understand the pathogenesis of VCP disease because they target the autophagy cascade and its intermediates at various locations (Fig 4A). Rapamycin, a key modulator of the mammalian Target of Rapamycin (mTOR) pathway has shown neuroprotection properties in several neurodegenerative diseases, including Alzheimer's disease, Parkinson's disease, Huntington's disease and spinocerebellar ataxia type 3 [71, 72, 85]. Rapamycin functions by inhibiting mTOR whose activation inhibits autophagy [86]. The accumulation of damaged proteins and the failure of autophagy clearing is a hallmark of VCP-associated diseases; therefore, we hypothesized that Rapamycin treatment may show some benefit. Here, we treated our cells with 10 μM Rapamycin for 24 hours and demonstrate significant reduction in the ‘classic’ VCP pathology markers TDP-43, LC3 and p62/*SQSTM1*, while mTOR activity was slightly diminished in VCP when compared to untreated patient samples (Fig 4B–4D). These results were confirmed by Western blot and densitometry (Fig 4G and 4H). Perifosine inhibits mTOR signaling through a different mechanism than classical mTOR inhibitors such as Rapamycin. Perifosine is an alkylaphospholipid, which induces cell cycle arrest and apoptosis through the inhibition of the serine-threonine protein kinase (Akt) also known as protein kinase B [73]. Several publications have shown that Akt and VCP interact and that VCP is a target of Akt signaling [87, 88], therefore we hypothesized that inhibition of Akt may be beneficial for VCP disease. In this report, we examined the effects of Perifosine by treating our cells (80 μM) and showed reduction in the “classic” VCP pathology markers TDP-43, LC3 and p62/*SQSTM1* when compared to untreated patient samples (Fig 4B, 4C and 4E). These results were confirmed by Western blot and densitometry with p<0.001 (Fig 4G and 4H).

**Fig 5:** Drug screening with autophagy inhibitors chloroquine, Spautin-1, and MHY1485 shows in patient VCP iPSC-derived myoblast lineages. (A) Untreated differentiated control and (B) untreated patient derived myogenic lineages. Patient derived myogenic lineage were treated with either (C) chloroquine (10 μM), (D) Spautin-1 (10 μM) or (E) MYH1485 (2 μM) for 24 hours. Subsequently, cells were stained with TDP-43, LC3 or p62/*SQSTM1* antibodies. Representative merged overlay images of stained iPSC with DAPI. Scale: Bar = 25 μm. White dotted lines represent areas of increased or decreased expressions. (F) Western blot analysis of iPSC-derived control and patient myoblasts probed against TDP-43, LC3-I/II, and p62/*SQSTM1* antibodies. GAPDH was used as a positive loading control. (G) Densitometry analyses from Western blot. Black dotted line indicates expression over baseline control sample.

Furthermore, we examined the effects of AT101, an orally available and well-tolerated natural BH3-mimetic that activates Bax and also induces mitochondrial Smac release in our *in vitro* model [75]. Here, we treated our cells with 10 μM AT101 and show reduction in VCP pathology marker TDP-43 and less so autophagy markers LC3 and p62/*SQSTM1* when compared to untreated patients (p<0.001) (Fig 4B, 4C, 4F, 4G and 4H).

Chloroquine is a lysosomotropic agent that prevents endosomal acidification [89]. Chloroquine inhibits autophagy as it raises the lysosomal pH, which leads to inhibition of both fusion of autophagosome with lysosome and lysosomal protein degradation [90, 91]. To uncover if chloroquine could reduce VCP pathology by inhibiting the formation of autolysosome, thought to be the “classic” vacuole associated with VCP disease, we treated our cells with 10 μM of chloroquine. Herein, we show chloroquine has no effect on VCP pathology markers TDP-43, LC3 and p62/*SQSTM1* when compared to untreated patient myoblasts (Fig 5A–5C). These results were confirmed by Western blot and densitometry (Fig 5F and 5G). Spautin-1 inhibits the activity of two ubiquitin-specific peptidases, USP10 and USP13, causing an increase in proteasomal degradation of class III PI3 kinase complexes, which have been shown to regulate autophagy [78]. To uncover if Spautin-1 could reduce VCP pathology by inhibiting autophagy downstream of Akt and mTOR we treated our cells with 10 μM Spautin-1. We found Spautin-1 had no effect on VCP pathology markers TDP-43, LC3 and p62/*SQSTM1* when compared to the untreated patient myoblasts (Fig 5A, 5B and 5D). These results were confirmed by Western blot and densitometry (Fig 5F and 5G). MHY1485 is an mTOR activator that potently inhibits autophagy by suppression of fusion between autophagosomes and lysosomes [79]. To uncover if MHY1485 could reduce VCP pathology by inhibiting autophagy by inducing mTOR we treated our cells with 2μM MHY1485. In this report, we show MHY1485 has no effect on VCP pathology markers LC3 and p62/*SQSTM1* when compared to untreated patient myoblasts (Fig 5A, 5B and 5E), however, TDP-43 was seen to be expressed correctly in the nucleus (Fig 5A, 5B and 5E). Although, spatial expression of TDP-43 was corrected, interestingly Western blot revealed its overexpression in our patient cells treated with MHY1485 (Fig 5F and 5G). LC3 and p62/*SQSTM1* overexpression levels were confirmed by Western blot and densitometry (Fig 5F and 5G).

## Discussion

Human induced pluripotent stem cells (hiPSCs) represent a versatile model system for studying diseases that affect a number of organs. When given the proper stimuli, hiPSCs can be differentiated into a number of desired cell types and tissues. Moreover, the consistency, expandability, and purity of the hiPSCs provide a valuable tool to screen and test drugs *in vitro*. Therefore, developing robust iPSC models of both rare and common disorders is an excellent option for those diseases requiring poorly accessible and/or limited availability tissue samples. Due to the pleiotropic nature of VCP disease, we recently established iPSC lines to elucidate the pathobiology and cellular and molecular mechanisms underlying this disease [55]. In the present study, we report the differentiation of VCP disease-specific hiPSCs into a myogenic lineage for the discovery of the underlying molecular mechanisms and the development of a drug-screening assay offering the significant possibility to intervene in the early stages of the disease. Ultimately, knowledge of the cellular and molecular signaling pathways affected by VCP mutations provides future promise in the development, assessment, and clinical application of pharmacological and gene therapies to prevent or slow down the progression of VCP disease.

We previously reported differentiation and characterization of VCP patient hiPSCs into a neural lineage [55]. These differentiated neural cells showed all the typical hallmarks of VCP pathology, including increased p62/*SQSTM1*, LC3-I/II and TDP-43. Inclusion body myopathy (IBM) is the most common feature present in 80–90% of affected VCP patients [5, 31]. Typically, the progressive muscle weakness rapidly advances resulting in patient mortality from cardiomyopathy or respiratory failure between approximately 40–60 years of age. The differentiation of human iPSCs into skeletal muscle cells has been challenging with methods ranging from serial media changes to viral infection of myogenic genes such as Pax7 [47, 64, 68]. Of note, an interesting observation we made was that staining with early myogenic precursor markers such as MYF-5, desmin, and Pax7 illustrated increased expression from Day 21, and they are still expressed at Day 50. Late myogenic markers (skeletal markers), such as MyoD and MYH2 were expressed by Day 50, however, not observed at earlier time points. However, a literature search suggested that Pax7 was expressed in the cytoplasm during different cell cycle stages and development [92, 93]. We hypothesize that these cells, aptly named myogenic lineage cells are not fully differentiated yet. However, we do believe they are suitable for our purpose of drug screening as they do display ‘classic’ VCP-associated disease pathology features. The reduced desmin organization and reduced MyoD expression are likely due to these cells not reaching full maturity.

To the best of our knowledge, this is the first article to fully differentiate patient-derived hiPSCs into a myogenic lineage modeling VCP-associated myopathy. These cells are 92% positive for CD56+ (myogenic markers) and mesenchymal stem cell markers (MSC+). Notably, we used these myogenic lineages to characterize the phenotypical features observed in humans. VCP disease muscle pathology is characterized by the presence of rimmed vacuoles, ubiquitin and TDP-43 positive inclusions and increased autophagy markers p62/*SQSTM1* and LC3 indicating a potentially dysfunctional autophagy pathway. Autophagy plays an important role in degrading defective organelles. Recent studies have shown that p62/*SQSTM1* interacts with the autophagic effector protein LC3-I/II to mediate the autophagic uptake of aggregated proteins. Previous researchers have shown that expression of VCP disease mutant proteins results from autophagosome accumulation and that these autophagosomes fail to mature into autophagolysosomes and degrade LC3; indicating autophagy is impaired in VCP disease [94]. Thus, we characterized the autophagy cascade and observed that the differentiated VCP myogenic lineage demonstrated a significant increase in the expression of p62/*SQSTM1*, LC3-I/II, and ubiquitin in comparison with the control myogenic lineage. There was also translocation of TDP-43 from the nucleus to the cytoplasm, another hallmark of VCP pathology thus suggesting that this patient derived myogenic lineage displays the typical of VCP disease pathology.

In the present study, we also examined the development of a rapid drug-screening assay to understand the true interactions of the underlying molecular mechanisms of VCP disease and how to target them in hopes to discover potential treatments for VCP disease. Our work as well as work from others indicating dysfunctional autophagy as the instigator of VCP muscle pathology led us to use our drug screening assay to target the autophagy pathway with potent inhibitors and activators [5, 30, 33, 83, 94].

Firstly, we investigated the activation of autophagy by treating our differentiated cells with autophagy stimulators Rapamycin, Perifosine, or AT101 [71–73, 75]. Rapamycin a key modulator of the mammalian Target of Rapamycin (mTOR) pathway has shown significant promise and neuroprotection in Alzheimer's disease, Parkinson's disease, Huntington's disease and spinocerebellar ataxia type 3 [71, 72, 85]. Rapamycin associates with mTORs intracellular receptor FKBP12 [95]. The FKBP12-rapamycin complex binds directly to the FKBP12-Rapamycin Binding (FRB) domain of mTOR, inhibiting its activity [95]. mTOR activation inhibits autophagy, however it simultaneously stimulates protein synthesis and cell growth which can result in accumulations of damaged proteins and organelles [86]. The accumulation of damaged proteins and the failure of autophagy clearing is a ‘hallmark’ of VCP disease and we hypothesized that Rapamycin treatment may ameliorate the dysfunctional autophagy cascade as it is upstream of VCP involvement in autophagy. Treatment with 10 μM of Rapamycin for 24 hours showed a reduction in the “classic” VCP pathology markers TDP-43, LC3 and p62/*SQSTM1* when compared to untreated patient, mirroring untreated control. Several publications have now shown that serine-threonine protein kinase (AKt) also known as protein kinase B and VCP interact and that VCP is a target of Akt signaling. Vandermoere *et al*. (2006) identified VCP as an essential target of Akt signaling and demonstrated that Akt and VCP co-immunoprecipitated and co-localized under Akt activation in MCF-7 breast cancer cells. In addition, they identified Ser-351, Ser-745, and Ser-747 as Akt phosphorylation sites on VCP via site-directed mutagenesis [87, 88]. We, therefore, hypothesized that inhibition of Akt may be beneficial for VCP disease. Perifosine is an alkylaphospholipid which induces cell cycle arrest and apoptosis through the inhibition of Akt [73]. mTOR is a target for Akt, the activation of which suppresses autophagy. In the event of ER stress such as in VCP disease, mTOR is innately downgraded to suppress protein production. All treatments with autophagy activators result in further reduction in mTOR, we hypothesize that by mechanistically reducing protein production mTOR inhibitors can improve VCP disease pathology. Perifosine has also been shown to exhibit anti-cancer properties, in bladder cancer, hepatocellular carcinoma and lung cancer [73, 96–98]. Treatment with 80 μM Perifosine showed reduction in the “classic” VCP pathology markers TDP-43, LC3I/II and p62/*SQSTM1* when compared to untreated patient, mirroring the untreated controls. Our last autophagy inducer, AT101, is an orally available and well-tolerated natural BH3-mimetic that activates Bax and also induces mitochondrial Smac release [75]. AT101 has shown anti-tumor activity as a single agent and in combination with standard anticancer drugs in a variety of tumor models [74]. We hypothesize that as AT101 works downstream of both Rapamycin and Perifosine, it may be more effective in ameliorating VCP pathology. We found treatment with 10 μM AT101 showed a reduction in VCP pathology markers TDP-43, LC3 and p62/*SQSTM1* when compared to untreated patient, mirroring untreated control. The results from these drug studies suggest that autophagy modulation, in particular autophagy activation agents, may be beneficial for patients suffering from VCP disease myopathy.

Secondly, we investigated the inhibition of autophagy by treating our differentiated cells with autophagy inhibitors chloroquine, Spautin-1 and MHY1485. Chloroquine is a lysosomotropic agent that prevents endosomal acidification [89]. Chloroquine inhibits autophagy by raising the lysosomal pH, which leads to inhibition of both fusion of autophagosome with lysosome and lysosomal protein degradation [90, 91]. Herein, we demonstrate chloroquine has no effect on VCP pathology markers TDP-43, LC3 and p62/*SQSTM1* when compared to untreated patient. Our second treatment was with Spautin-1 which promotes the degradation of Vps34 PI3 kinase complexes by inhibiting two ubiquitin specific peptidases, USP10 and USP13, which target the Beclin1 subunit of Vps34 complexes. Since USP10 mediates the de-ubiquitination of p53, regulating de-ubiquitination activity of USP10 and USP13 by Beclin1 provides a mechanism for Beclin1 to control the levels of p53. By this mechanism, Spautin-1 increased cancer cell death in the setting of nutrient deprivation when autophagy would normally act as a survival mechanism in these metabolically stressed cells [78]. We discovered treatment with Spautin-1 (10 μM for 24 hours) had no effect on VCP pathology markers TDP-43, LC3 and p62/*SQSTM1* when compared to untreated patient. Lastly we tested MHY1485, which is an mTOR activator that potently also inhibits autophagy by suppression of fusion between autophagosomes and lysosomes [79]. To uncover if MHY1485 could reduce VCP pathology, by inhibiting autophagy, by inducing mTOR, we treated our cells with MHY1485. We hypothesized that it could have a negative effect, as previous studies showed MHY1485 leads to the accumulation of LC3-I/II and enlargement of the autophagosomes in a dose- and time- dependent manner [79]. Interestingly, we demonstrated that treatment with MHY1485 (2 μM for 24 hours) had a modest beneficial effect on VCP pathology with a decrease in markers LC3 and p62. Also, TDP-43 was observed to be expressed in the correct location (nucleus), mirroring our control cells. However, although spatial expression of TDP-43 was corrected, Western blot revealed it is still overexpressed in our patient cells treated with MHY1485. Future studies with varying MHY1485 doses and treatment times will be needed to uncover if MHY1485 could be beneficial for VCP patients. Future in-depth studies into the autophagy and mitophagy cascades, cell survival and animal studies to investigate the effects of these drugs on muscle function and structure need to be completed.

## Summary and conclusions

Herein, we report the successful differentiation of VCP patient specific hiPSCs into myoblasts exhibiting phenotype and dysfunction characteristics of typical VCP disease autophagy and thus providing a novel platform for a rapid drug screening. Evaluation of the ameliorative effects of several autophagy modifiers using these cells as a drug-screening platform revealed that some autophagy modulators may hold promise for VCP disease myopathy. The VCP hiPSC model system offers a unique platform in understanding the underlying pathophysiology molecular mechanisms and vistas in improving muscle integrity and/or slowing down the progression of muscle wasting in patients with VCP and related neurodegenerative diseases.
